# Unilateral Sciatic Nerve Crush Induces White Blood Cell Infiltration of the Contralateral Nerve

This article has been retracted.

**DOI:** 10.1155/2022/1101383

**Published:** 2022-03-29

**Authors:** Jia Cheng, Lingtao Ding, Minlie Yang, Yugang Zhu, Zaiqiu Gu, Guozhong Lv

**Affiliations:** Department of Burn and Plastic Surgery, Affiliated Hospital of Jiangnan University, Wuxi, Jiangsu, China

## Abstract

Nerve injury leads to the accumulation of white blood cells derived from the bone marrow in the lesioned nerve, but it is still unknown whether there are similar responses in unlesioned nerves. To address this question, sciatic nerves of mice expressing enhanced green fluorescent protein (EGFP) in their bone marrow were crushed unilaterally to observe the invasion of bone marrow-derived cells into the contralateral unlesioned nerve. Two days after surgery, EGFP^+^ cells began to infiltrate both the damaged and undamaged nerves. These cells gradually amplified to the highest point within 14 days and slowly lowered. In ipsilateral (lesioned) and contralateral (unlesioned) nerves, the time course of infiltration of EGFP^+^ cells was similar, but the magnitude was much less for the unlesioned one. Through CD68 staining, some cells were identified as macrophages. Transmission electron microscopy revealed slight demyelination and phagocytosing macrophages in the contralateral nerve. The data showed that infiltration by white blood cells is a response to nerve injury, even in uninjured nerves.

## 1. Introduction

Peripheral nerve degeneration after an injury is characterized by the breakdown of axons and myelin sheaths, glial cell proliferation, blood-nerve barrier compromise, and dramatically, phagocytosis by macrophages of Schwann cells in the distal nerve which is called Wallerian degeneration [1–4]. There are two kinds of macrophages within the Wallerian degeneration: hematogenous macrophages derived from the bone marrow and resident endogenous macrophages. Cámara-Lemarroy et al. [5] and Koltzenburg et al. [6] have found that, in addition to the phagocytosing axon and myelin remnants, macrophages could promote proliferation of Schwann cells and fibroblasts and release neurotrophic factors and cytokines [7, 8].

The nervous system of mammals has a high degree of bilateral symmetry [9]. There is a wide range of examples in which unilateral interventions produce bilateral effects [10–12]. In the center nerve system, unilateral injury to the lateral fimbria resulted in bilateral gliosis in the septum and hippocampus. Some cellular and molecular changes in the contralateral DRG and sciatic nerve after unilateral peripheral nerve injury have also been described [9, 13]. There is no study showing whether there are changes or not in the contralateral sciatic nerve after unilateral injury, nor has any report discussed the differences between cell infiltration patterns in the contralateral nerve compared with the ipsilateral side.

The aim of this research was to find out whether white blood cells derived from the bone marrow invade the contralateral sciatic nerve after unilateral injury and analyze the pattern of such infiltration. To track bone marrow-derived cell infiltration, we utilized irradiated bone marrow chimera mice that expressed EGFP in all bone marrow-derived cells [5, 14]. Preparations were counterstained with an antiserum against CD68, a marker of macrophages, to visualize hematogenous macrophages infiltration from the systemic circulation. Two days, sciatic nerves were extracted at 1, 2, 4, 8, 12, and 30 weeks following the crush injury and tested through immunofluorescent staining and transmission electron microscopy.

## 2. Materials and Methods

### 2.1. Bone Marrow-Irradiated Chimeric Mice

The Animal Ethics Committee of the Chinese Academy of Medical Sciences and Peking Union Medical College approved all experimental methods. As previously stated, chimeric mice were created [13–15]. On a C57BL/6J genetic background, EGFP transgenic mice expressing the enhanced green fluorescent protein gene were utilized (Model Animal Research Central of Nanjing University, Nanjing, China). 9 Gray was used to irradiate wild-type C57BL/6J mice (Shanghai SLAC Laboratory Animal Co., Ltd., Shanghai, China). Following that, donor bone marrow cells were extracted from the long bones of EGFP^+^ mice, and 8106 cells were injected into the tail vein by injection. Only chimeras with >95 percent EGFP^+^ leukocytes were used for additional studies after 3 months. Fluorescence microscopy was used to measure the percentage of EGFP^+^ leukocytes in chimera mice.

### 2.2. Sciatic Nerve Injury and Tissue Processing

Intraperitoneal injection of ketamine/xylazine was used to deeply anesthetize mice. Only the epineurium remained intact after the right sciatic nerve was crushed for 15 seconds distal to the sciatic notch using forceps. Six mice from each group were allowed to survive for 2 days, 1, 2, 4, 8, 12, and 30 weeks after crush injury. Sciatic nerves were then extracted and fixed for 2 hours in a 10% sucrose solution with 4% paraformaldehyde, then submerged in a 30% sucrose solution at 4°C overnight. Samples were embedded in optimal cutting temperature compound (OCT) for frozen sections, and 10 mm thick cryosections were produced with a cryostat-microtome (Thermo, Cheshire, USA). The contralateral transverse sections were obtained at a site that was roughly comparable to the crash damage.

### 2.3. Immunofluorescence Analysis

The slides were rinsed with PBS and masked in a solution that contains 10% goat serum at ambient temperature, followed by an incubation period at 4°C with rat anti-CD68 antibody (1 : 250, Serotec, Oxford, UK). Finally, the sections were treated with Alexa Fluor 555-donkey anti-rat IgG for 45 minutes at 37°C (1 : 1000, Invitrogen, Carlsbad, USA). 4′,6-diamidino-2-phenylindole (DAPI; 1 : 500, Invitrogen) was used to counterstain the nuclei for 30 seconds. A confocal microscope was used to capture the fluorescent pictures (Leica SP5, Germany). The intensity of immunofluorescence staining was measured using the Image-Pro Plus 6.0 software (Media Cybernetics, USA) to calculate the integrated optical density (IOD) of positive expression from six randomly selected sections, as described previously [16].

### 2.4. Transmission Electron Microscopy

Sciatic nerves were preserved in 2% glutaraldehyde for 2 hours at 4°C then in 1% osmic acid (diluted with PBS) for 2 hours at 4°C. Sciatic neurons were dehydrated to use a graded series of alcohol solutions in the sequence shown below after being washed with PBS. The sciatic nerve cells were washed with PBS and dehydrated with the gradient series of alcohol solution as shown in the following sequence: 30%–50%–70% and 80%–95%–100% alcohol 10 min each. After that, the alcohol was replaced with epoxypropane for 10 minutes, followed by epoxy resins 618 and epoxypropane (1 : 1) for 2 hours, and then the mixture was heated to 60°C for 48 hours. Using an LKB-V ultramicrotome (LKB ProdukterB, Stockholm; Sweden), semithin sections (1 mm thickness) and ultrathin sections (50 nm thickness) were cut, stained with lead citrate, and examined under CM-120 transmission electron microscopy (Philips, Netherlands).

### 2.5. Statistical Analysis

All of the data were presented as means with standard deviations (SD). When applicable, values were established using paired *t*-tests between two groups and one-way analysis of variance (ANOVA) among three or more groups using SPSS version 19.0 (Chicago, IL, USA) for quantitative comparison and analysis. Statistical significance was defined as a *P* value of less than 0.05.

## 3. Results

### 3.1. Bone Marrow-Derived EGFP^+^ Cells Invade the Contralateral Uninjured Nerve

Very few EGFP^+^ cells were detected in normal sciatic nerve (Figure 1(a), control). To observe whether the uninjured nerve had any changes of bone marrow-derived EGFP^+^ cells after unilateral nerve crush, both nerves were harvested at 2 days and 1, 2, 4, 8, 12, and 30 weeks after injury. Similar to the injury site, on day 2, EGFP^+^ cells began invading the contralateral neuron, which steadily grew to a peak at 2 weeks before gradually decreasing (Figure 1(a)). Interestingly, EGFP^+^ cells of the injured side dropped to a normal level within 12 weeks; but on the contralateral side, they were still elevated (Figure 1(b)). In addition, most EGFP^+^ cells were arranged in a longitudinal direction within the entire nerve (Figure 2). Contralateral nerve segment EGFP^+^ cell infiltration patterns were identical to ipsilateral nerve segment infiltration patterns. The number of EGFP^+^ cells in contralateral nerve segments, on the other hand, was lower than in ipsilateral nerve segments. The contralateral: the ipsilateral ratio was around 1 : 11.5 at 2 weeks (Figure 1(b)).

### 3.2. Variation of Macrophages on the Contralateral Side

Macrophages are the crucial effector cells in neuropathies [17]. To identify and localize bone marrow-derived macrophages, EGFP autofluorescence was combined with a CD68 antibody. In normal sciatic nerve, very few resident macrophages (EGFP^−^/CD68^+^) were observed in either nerve (Figure 3(a), Control). Two days, 1, 2, 4, 8, 12, and 30 weeks after crush injury, numerous hematogenous macrophages (EGFP^+^/CD68^+^) as well as resident macrophages were present in the injured nerve (Figure 3(a)), and hematogenous macrophages increased more obviously than resident macrophages (Figure 3(b)). On the contrary, on the contralateral side, only a few EGFP^+^ cells were macrophages (Figure 3(a)), and hematogenous macrophages were significantly less than resident macrophages (Figure 3(b)). When the total number of EGFP^+^ cells and macrophages (Total M) in the crush-injured nerve was compared to the contralateral nerve, the total number of EGFP^+^ cells and macrophages (Total M) was found to be significantly higher in the crush-injured nerve (Figures 1(b), 3(b), and 3(c)).

### 3.3. Ultrastructure of the Contralateral Nerve

After nerve injury, macrophages penetrate the Schwann cell basal lamina to reach and phagocytose the myelin. To assess whether there was the same phenomenon in the contralateral uninjured nerve, we examined the nerves after 2 weeks of crush injury by electron microscopy. The results demonstrated that most myelin sheaths were normal and complete in the contralateral nerve (Figure 4(a)). However, typical degenerative Schwann cell alterations were also observed (Figures 4(b) and 4(c)). In addition, motile macrophages with elongated cytoplasmic processes located outside the Schwann cell basal lamina were noticed to be sparsely distributed (Figure 4(c)). Some macrophages with lipid droplets and end products of myelin-degradation were presented as phagocytosing macrophages (Figure 4(c)). These data provided strong evidence that the contralateral nerve also undertook slight demyelination and inflammatory reaction after unilateral sciatic nerve crush.

## 4. Discussion

When the peripheral nervous system is damaged, a complicated cellular immune response emerges. Neutrophils are the first immune cells to assemble in the distal stump, and they do so within 8 hours. Hematogenous macrophages take over as the main leukocyte population as a result. In addition, local macrophages have been discovered to have a role in Wallerian degeneration. In peripheral nerves, resident macrophages makeup 2–9 percent of total cells and are known to be phagocytic. To date, whether hematogenous immune cells are recruited into the contralateral sciatic nerve has never been investigated. Our study corroborated that the infiltration by white blood cells in one nerve also appears in the contralateral uninjured nerve at the same time [18].

In our study, bone marrow chimeric animal models were used to detect bone marrow-derived cells. Together with the colocalization of CD68, resident and hematogenous macrophages could be separated from other cells easily. In our mice, rapid EGFP^+^ cell infiltration and macrophages activation were found in the injured nerve. A similar time course of infiltration of EGFP^+^ cells was also seen on the contralateral side, but many fewer infiltrating cells were seen. Interestingly, in the contralateral nerve, only a few bone-derived marrow-derived cells were EGFP^+^/CD68^+^, which was in sharp contrast to the injured nerve. This may be because other hematogenous immune cells have a more important role than macrophages in the contralateral response. These available data indicated that macrophage reaction patterns had a close relationship with the severity of damage in the peripheral nerve system. Only under the circumstance of more severe damages, an additional influx of macrophages is initiated, together with resident macrophages to exert their functions [19].

Macrophages will efflux out of the lesioned Schwann cell basal lamina and nerve once phagocytosis is done, allowing for effective repair and regeneration [18, 19]. In addition, Fry et al. [20] have demonstrated that the presence of new myelin promotes macrophage outflow from the Schwann cell basal lamina and impacts their final exit from the lesioned nerve. In our experiment, EGFP^+^ cells moved out of the contralateral nerve more slowly than from the injured nerve. This might be due to less newly synthesized myelin, so fewer signals were sent to EGFP^+^ cells to migrate out of the nerve [21].

One explanation for contralateral involvement is that the lesion-induced signals from the spinal commissural interneurons where hematogenous macrophages and the retrograde signal could be transported from the injury site during Wallerian degeneration could induce cellular and molecular changes in the contralateral side. Another possible reason is the blood transmission of the damage-induced signals to the contralateral side. During Wallerian degeneration, the blood-nerve barrier becomes more permeable for large molecules. Therefore, blood flow might deliver factors from the injured nerve to the contralateral nerve which could initiate the invasion of EGFP^+^ cells. However, some limitations and shortcomings of our research still need to be improved in our further experimentation, such as the exact mechanism responsible for contralateral involvement and how the contralateral nerve can get information from the injured nerve remain unknown. Our data describe for the first time unilateral sciatic nerve crush induces white blood cell infiltration of the contralateral nerve. That is, is this increase in infiltration, and the associated slight disruption of myelin, a general response of all peripheral nerves to local lesions, or a specific response to uninjured sciatic nerves [22]?

## 5. Conclusion

In this study, we concluded that an immunologically mediated hematogenous cells response could take place in the uninjured nerves, which had a similar infiltration trend with the injured side. Studies focusing on the contralateral nerves may also have implications for our comprehensive understanding of peripheral nerve pathophysiology [23].

## Figures and Tables

**Figure 1:** EGFP^+^ cells infiltration in the contralateral and ispilateral sciatic nerves after unilateral injury. (a) EGFP^+^ cells in the contralateral (contra) and ispilateral nerves (Ipsi). (b) Quantification of EGFP^+^ cells at different time points. Control: normal sciatic nerve. Bar = 100 *μ*m. ^*∗*^*P* < 0.05.

**Figure 2:** EGFP^+^ cells distribution in the whole entire contralateral nerves. The longitudinal distribution of EGFP^+^ cells within contralateral and ispilateral nerves 1 week, 2 weeks, and 4 weeks after injury. Bar = 500 *μ*m.

**Figure 3:** Localization of endogenous and hematogenous macrophages at different time points. (a) CD68 staining (red) and EGFP^+^ cells within the contralateral and ispilateral nerves. (b) Quantification of macrophages at different time points. Total M: total macrophages; EGFP^−^/CD68^+^ M: endogenous macrophages (arrowhead, red); EGFP^+^/CD68^+^ M: hematogenous macrophages (arrow, yellow). Bar = 100 *μ*m. ^*∗*^*P* < 0.05.

**Figure 4:** Ultrastructure of the contralateral sciatic nerves 2 weeks after injury. (a) Normal and complete myelin sheaths in the contralateral nerve. Demyelinating phenomenon ((b), arrow) and active macrophages with elongated cytoplasmic processes and deris filled the cytoplasm ((c), arrowhead) were present in the contralateral nerve. Bar (a) = 10 *μ*m. Bar (b, c) = 2 *μ*m.

## Data Availability

The data used to support this study are available from the corresponding author upon request.
